This article has been retracted.

# Inactivation of MAP kinase signalling in Myc Transformed Cells and Rescue by LiCl inhibition of GSK3

**DOI:** 10.1186/1476-4598-4-13

**Published:** 2005-04-05

**Authors:** Osama Al-Assar, Dorothy H Crouch

**Affiliations:** 1 Biomedical Research Centre, University of Dundee, Ninewells Hospital and Medical School, Dundee DD1 9SY, UK; 2 Institute for Cancer Studies, Division of Genomic Medicine, Medical School, University of Sheffield, Beech Hill Road, Sheffield S10 2RX, UK

## Abstract

c-Myc oncogene is an important regulator of cell cycle and apoptosis, and its dysregulated expression is associated with many malignancies. Myc is instrumental in directly or indirectly regulating the progression through the G1 phase and G1/S transition, and transformation by Myc results in perturbed cell cycle. Also contributory to the control of G1 is the Ras effector pathway Raf/MEK/ERK MAP kinase. Together with GSK3, ERK plays an important role in the critical hierarchical phosphorylation of S62/T58 controlling Myc protein levels. Therefore, our main aim was to examine the levels of MAPK in Myc transformed cells in light of the roles of ERK in cell cycle and control of Myc protein levels. We found that active forms of ERK were barely detectable in v-Myc (MC29) transformed cells. Furthermore, we could only detect reduced levels of activated ERK in c-Myc transformed cells compared to the non-transformed primary chick embryo fibroblast cells. The addition of LiCl inhibited GSK3 and successfully restored the levels of ERK in v-Myc and c-Myc transformed cells to those found in non-transformed cells. In addition, LiCl stabilised Myc protein in the non-transformed and c-Myc transformed cells but not in v-Myc transformed cells. These results can provide an important insight into the role of MAPK in the mechanism of Myc induced transformation and carcinogenesis.

## Background

The c-Myc oncogene is one of the most frequently dysregulated genes in human tumours. Myc was originally identified as the cellular homolog of the transforming part of the viral isolate MC29 [1]. The c-Myc oncogene is a member of the basic-helix-loop-helix-leucine-zipper transcription (bHLH-ZIP) factors, which are essential for different cellular processes [2]. Paradoxically, c-Myc promotes both cell cycle progression and apoptosis under low serum condition [3,4]. c-Myc regulates the cellular processes by controlling a large number of target genes [5,6] through heterodimerization with its biological partner Max [7-9]. The abundance of the Myc-Max heterodimer is effectively controlled by the short lived Myc protein [10]. The Myc protein is under tight and complex control mechanisms [11].

Critical phosphorylation events determining the protein half life occur in Myc homology box I (aa45-aa65) [10]. These detrimental events involve the hierarchical phosphorylation of S62 and T58 by ERK1/2 MAPK and GSK3β, respectively [12]. It is widely accepted that these kinases are involved in the phosphorylation events at these residues although other reports question the role of MAPK [13]. These two kinases are part of two different Ras effector pathways. The presence of different Ras isoforms provides for selective activation of specific Ras effector pathway, although this can only be shown in vivo [14]. It has been reported that PI-3 kinase is most effectively activated by M-Ras and R-Ras and to a less extent by H-Ras [15,16]. On the other hand, Raf-1 is most effectively activated by K-Ras [17,18]. This selective activation of different Ras effector pathways has opposing effects on Myc controlled functions. Whereas the activation of Raf fails to suppress Myc induced apoptosis, the activation of PI-3 Kinase can effectively suppress it [19]. A key component of the PI3-kinase/Akt (PKB) pro-survival pathway is GSK3 [20], whereas the active phosphorylated form of ERK1/2 MAPK is a downstream signal in the signalling cascade Ras/Raf/MEK [21].

The ERK1/2 MAPK is one of three major MAPK signalling pathways, which also includes JNK/SAPK and p38 kinase. Constitutive activation of MEK/ERK has been reported in cancer cells [22,23], with a possible role in cell transformation and oncogenesis [24]. The constitutive activation of MAPK ERK1/2 could be linked to the mitogen independence reported for oncogenes like Ras [25], Raf [26], Jun [27] and Myc [4]. Therefore, one of the aims of this study was to examine the status of active ERK2 in Myc transformed chick embryo fibroblasts (CEF), the ideal model for Myc induced transformation.

Our second aim was to examine the possibility of a cross talk between ERK2 and GSK3 in Myc transformed fibroblasts using LiCl to inhibit GSK3. Reports on signalling between GSK3 and ERK1/2 are very scarce. Nonetheless, a recent report has demonstrated that GSK3β was a natural activator of the JNK/SAPK pathway [28]. Furthermore, it has been demonstrated that GSK3β could be phosphorylated on Ser9 and therefore inactivated by ERK1/2 mediated pathways, mainly through p90^rsk ^but also through a novel mechanism downstream of ERK1/2 [29]. These findings need to be verified in transformed phenotype.

## Results and Discussion

We have found that v-Myc (MC29) transformed fibroblasts have almost non-detectable active ERK2 (Figure 1A). A control experiment using the SFCV vector without an insert was performed in parallel with every experiment to exclude any effect for the transfection procedure. Cells transfected with the control vector gave identical results to the non-transfected control CEF cells. The addition of 100 mM LiCl was very successful in restoring (not fully) the levels of active ERK2 in v-Myc transformed fibroblasts to those found in non-transformed fibroblasts within the time scale of the experiment. The barely detectable basal levels of phosphorylated ERK2 in v-Myc transformed fibroblasts showed an increase after the addition of LiCl at the earliest time point of 20 minutes (31% of basal levels in non-transformed control CEF). These levels were almost completely restored to the levels found in non-transformed CEF after 80 minutes (83% of basal levels in non-transformed control CEF).

**Figure 1:** **The effect of LiCl on the levels of active ERK in Myc transformed and non transformed fibroblasts. (A) **A time course for the effect of LiCl on the levels of active ERK2 in v-Myc transformed fibroblasts (panel 1). Total ERK levels were not affected and were used as a loading control (panel 2). Panel 3 is a graphical representation of the ERK2 levels in Li^+ ^and K^+ ^treated v-Myc cells after normalisation to ERK2 levels in non-transformed control CEF (identical to CEF transfected with empty vector) growing under normal conditions. **(B) **A time course for the effect of LiCl on the levels of active ERK2 in c-Myc transformed fibroblasts (panel 1). Total ERK levels were not affected and were used as a loading control (panel 2). Panel 3 is a graphical representation of the ERK2 levels in Li^+ ^and K^+ ^treated c-Myc cells after normalisation to ERK2 levels in non-transformed control CEF growing under normal conditions. **(C) **A time course for the effect of LiCl on the levels of active ERK2 in non-transformed control CEF (panel 1). Total ERK levels were not affected and were used as a loading control (panel 2). Panel 3 is a graphical representation of the ERK2 levels in Li^+ ^and K^+ ^treated cells after normalisation to ERK2 levels in non-transformed control CEF growing under normal conditions. The same pattern of expression was seen in several independent experiments for all the panels.

On the other hand, c-Myc transformed fibroblasts have shown attenuated but detectable active ERK2 levels compared to the non-transformed CEF. The addition of 100 mM LiCl fully restored the levels of active ERK2 to those found in non-transformed CEF (Figure 1B). The reduced basal levels of ERK2 in c-Myc transformed fibroblasts showed an increase at the earliest time point of 20 minutes (88% of basal levels in non-transformed control CEF) after the addition of LiCl and were comparable to the levels seen in the non-transformed CEF after 60 minutes. In the non-transformed CEF, the addition of LiCl enhanced the levels of active ERK2 considerably (Figure 1C). The increase in the levels of active ERK2 in CEF after the addition of LiCl was detectable after 20 minutes (153% of basal levels in non-transformed control CEF) and peaked after 40 minutes (350% of basal levels in non-transformed control CEF).

In addition, adding 100 mM of LiCl increased the levels of inactive phosphorylated GSK3 α/β in a time dependent manner (Figure 2) in agreement with the pattern seen for the restored levels of active ERK2. We confirmed the activation of the pro-survival pathway PI3K signalling pathway after the addition of LiCl by the inhibition of apoptosis in Myc transformed fibroblasts (Figure 3). Compared to the KCl control, LiCl treatment resulted in 2.1, 3.6 and 2.4 fold reduced apoptosis in v-Myc, c-Myc and non-transformed control fibroblast cells, respectively. The different cell populations showed variable number of apoptotic cells after serum starvation. This is expected since v-Myc is a stronger inducer of proliferation and apoptosis than c-Myc [30,31]. Other researchers have also demonstrated that inhibition of GSK3 using LiCl was contributory to apoptosis inhibition[32]. Other GSK3 inhibitors can be used to further support these findings.

**Figure 2:** **The effect of LiCl on the levels of GSK3 in non-transformed fibroblasts. (A) **A western blot showing the levels of inactive or phosphorylated GSK3 α/β in non-transformed fibroblasts after the addition of Li^+ ^or K^+ ^salt control for the time points indicated. **(B) **A western blot showing the levels of phosphorylated and non-phosphorylated GSK3 α/β of the same samples in (A) above after stripping and re-probing of the blot with the appropriate antibody.

**Figure 3:** **The effect of LiCl on the apoptosis levels of serum starved Myc transformed and non-transformed fibroblasts. (A) **A graphical representation of the percentage of apoptotic v/c-Myc transformed and non transformed fibroblasts 17 hours after serum deprivation and addition of Li^+ ^or K^+^. The error bars are the standard error of three independent experiments. The total number of cells counted for each experiment was 50 cells. **(B) **&**(C) **Representative sections of Hoeschst 33258 stained c-Myc cells after K^+ ^and Li^+ ^treatment, respectively.

Similar to what we have observed in our Myc transformed cells, previous researchers have demonstrated that ERK1/2 activity was repressed in c-Raf-1 (Raf22W), v-Ha-Ras, and v-Src transformed cells by a single-specificity tyrosine phosphatase [33]. A more recent report has also demonstrated attenuated levels of ERK2 in v-Jun transformed CEF cells, which was attributed to inefficient signalling between Ras and Raf, and increased levels of MAPK phosphatase [34].

In light of the roles of ERK and GSK3 in Myc protein phosphorylation and stability, we investigated the effect of LiCl addition on Myc protein half life in c-/v-Myc transformed fibroblasts. Figures 4A and 4B show that the addition of LiCl results in dramatic stabilisation of Myc in the non-transformed and c-Myc transformed cells, respectively. Surprisingly, although endogenous Myc is hardly detectable in non-transformed CEF (t_1/2 _< 1 minute), it was 30 fold more stable after the addition of LiCl (Figure 4A). We verified this using immunoprecipitation (data not shown). In comparison, c-Myc protein was 4 fold more stable after LiCl treatment. Not surprisingly, both endogenous Myc in non-transformed control fibroblasts and exogenously expressed Myc in c-Myc transformed fibroblasts had similar half life values after the addition of LiCl (30 and 32 minutes, respectively). However, LiCl failed to further stabilise Myc in v-Myc transformed fibroblasts (Figure 4C). Myc protein half life was 40 minutes compared to 38 minutes in the control cells. Since MC29 v-Myc has T58>M (T61>M in chicken), we did not expect any effect for LiCl on Myc protein half life in these cells, although it was a necessary control. Other researchers documented a small effect for LiCl on Myc stability (2 fold) in immortalised cell lines [35]..

**Figure 4:** **Myc protein turnover after the addition of LiCl in Myc transformed and non transformed fibroblasts. (A) **Endogenous Myc protein in Li+ and K^+ ^treated non-transformed fibroblasts. This was identical to fibroblasts transfected with empty vector. Panel 1 is the scanned image of a western blot autoradiograph. Panel 2 shows the half life values of the Myc protein under the different conditions. CEF represents the non-transformed control fibroblasts **(B) **Turnover of the Myc protein in Li+ and K^+ ^treated c-Myc transformed fibroblasts. Panel 1 is the scanned image of a western blot autoradiograph. Panel 2 shows the half life values of the Myc protein under the different conditions. CEF represents the non-transformed control fibroblasts **(C) **Turnover of the Myc protein in Li^+ ^and K^+ ^treated v-Myc transformed fibroblasts. Panel 1 is the scanned image of a western blot autoradiograph. Panel 2 shows the half life values of the Myc protein under the different conditions. CEF represents the non-transformed control fibroblasts. The experiments were independently repeated three times and one representative experiment is shown.

We can conclude that LiCl has direct effects on the hierarchical phosphorylation of S62 and T58 (S65 and T61 in chicken) by controlling the levels of active ERK2 and GSK3, respectively. The results in this study show that this is important for the Myc half life in the non-transformed and c-Myc transformed fibroblasts but not in the v-Myc transformed cells. In this context, other researchers have found that S62 phosphorylation was necessary for Myc stabilization following Ras activation or serum stimulation[36].

## Conclusion

In this short communication we provided important findings about Myc induced transformation. The abrogation of active MAPK in Myc transformed cells can potentially provide an insight into the mechanism of Myc induced transformation. Clarification of the mechanism of ERK2 inactivation in Myc transformed CEF is needed. Furthermore, it is critical to examine the implications of the differences in active ERK2 levels between v-Myc and c-Myc transformed cells and the possible role this has in Myc induced transformation and protein stability. Last, we need to elucidate on the possibility of a cross-talk between GSK3 and ERK, as this could be a very important mechanism for controlling the Myc protein.

## Methods

### Cell Culture, Transfection and Inhibition Studies

Cell culture and transfection of the appropriate SFCV-Myc construct (10 μg) together with RCAN(A) helper (4 μg) into secondary CEF were performed as described previously [37]. A control experiment using the SFCV vector without an insert was used with every experiment as a transfection control. After G418 Neomycin selection (BDH, UK), cultures were expanded and used for the subsequent studies. At this stage, cells transfected with vectors containing either c-Myc or v-Myc were fully transformed as determined by anchorage independent growth and visible transformation characteristics, such as metamorphosis (data not shown). LiCl was added for 30 minutes at a final concentration of 100 mM to exponentially growing CEF, c-Myc or v-Myc cells before harvesting for western blotting. KCl was used in all the experiments as a salt control. For the Myc protein turnover studies, a protein synthesis inhibitor (emetine from Sigma, UK) was added 30 minute after the addition of either LiCl or KCL at a final concentration of 0.1 mM [38] for the indicated times shown in the figure.

### Apoptosis Induction and Measurement

Apoptosis was induced by incubating the cells in a medium containing 0.2% serum for 17 hours. Serum starvation for longer periods of time resulted in apoptosis in almost all of the v-Myc cell population. To measure the percentage of the apoptotic cells, the cell population was divided into adherent and suspended cells. The adherent cells were trypsinised, washed in 1× phosphate buffered saline (PBS) and fixated in ice cold 3:1 glacial acetic acid/methanol solution. Then, the cells were permealised at room temperature using a solution of 1× PBS/0.1% triton X-100 for 5 minutes. The cells were then stained in a solution of 2.5 μg/μl Hoeschst 33258 (Sigma, UK) in 1× PBS/0.1 % triton X-100 on ice and protected from light. After that, the cells were washed twice in 1× PBS/0.1% triton X-100, made adherent onto a slide using a cytospin, and viewed and counted under an epi-fluorescent microscope using a DAPI filter. We treated the suspended cells in exactly the same way with the exception that they did not need trypsinisation. To calculate the total number of apoptotic cells in both adherent and suspended cells, we used the following formula:



### SDS PAGE Western Blotting and Protein Half Life Measurement

Cell lysates were prepared by lysing cultures in SDS-sample buffer containing 1% SDS without bromophenol blue or mercaptoethanol. Protein concentration was measured using Micro BCA reagent (Pierce, UK) before loading onto 7.5% SDS-PAGE gels. Transfer to nitrocellulose and western blotting was performed essentially as described previously [37], except that incubation with the primary antibody was performed in 2.5% BSA in TBS-Tween20 for ERK western blots. Active phosphorylated ERK was detected using rabbit polyclonal antibodies (catalogue number 9101, New England Biolabs, UK) and total phosphorylated and non-phosphorylated ERK levels were detected using rabbit polyclonal antibody (catalogue number 71–1800, Zymed, UK). Inactive phosphorylated GSK3 α/β (Ser21/9) protein was detected using a rabbit polyclonal antibody (catalogue number 9331S, Cell Signaling Technology, UK) and phosphorylated and non-phosphorylated GSK3 α/β levels were detected using a rabbit polyclonal antibody raised against GSK3 β but detected both GSK3 α and β (catalogue number 9332, Cell Signaling Technology, UK). Full length Myc protein was expressed in our laboratory and was used to raise rabbit polyclonal antibodies against. To re-probe a blot, it was first submerged in a solution containing 100 mM 2-mercaptoethanol, 2% SDS and 62.5 mM Tris HCl pH 6.7 at 50°C for 1 hour, with agitation. Then, the blot was washed in a solution containing TBS/0.1% Tween20 for 10 minutes three times at room temperature. Last, the blot was blocked and probed as above with the appropriate antibody. Equal loading of lanes was determined by staining the polyacrylamide gel after transfer onto a nitrocellulose membrane in coomassie blue solution for 2 hours (50% methanol, 10% acetic acid, 0.25% coomassie blue R-250) and de-staining in a solution containing 10% methanol and 5% acetic acid for 4 hours. The different band intensities were analysed using the Kodak 1D image analysis software and then they were plotted on a linear graph for the ERK levels. For the calculation of the Myc protein half life, the densitometric values were plotted on a semi-logarithmic graph against time and then fitted to an exponential line. The half life of the protein was calculated from the equation:


